# Mathematical Modelling of Destabilization Stress Factors of Stable-Elastic Fixation of Distal Trans- and Suprasyndesmotic Fibular Fractures

**DOI:** 10.1155/2021/6607364

**Published:** 2021-11-09

**Authors:** Andriy Chuzhak, Vadym Sulyma, Lіubomyr Ropyak, Andrii Velychkovych, Vasyl Vytvytskyi

**Affiliations:** ^1^Ivano-Frankivsk National Medical University of the Ministry of Health of Ukraine, Halytska Str. 2, Ivano-Frankivsk 76018, Ukraine; ^2^Ivano-Frankivsk National Technical University of Oil and Gas, 15 Karpatska Street, Ivano-Frankivsk 76019, Ukraine

## Abstract

**Introduction:**

Specification of possible stress factors destabilizing the fibula stable osteosynthesis by the intramedullary nail with distal blocking and elastic fixation of distal syndesmosis by the thread with endobuttons by mathematical modelling of distal unstable ankle injuries. *Material and Methods*. We studied the thread tension during the combined stable-elastic fixation of unstable injuries of the ankle joint in cross-syndesmosis fractures of the fibula (B, C Danis–Weber classification), which includes a one-time stable minimally invasive fixation with the intramedullary nail and elastic fixation by the thread with endobuttons. We used a titanium alloy for the intramedullary nail and polyester for the thread. The deformed state was studied using the methods of mechanics.

**Results:**

A model of a fractured fibula blocked with the intramedullary nail and fixed with the elastic thread was developed. A formulation to specify the rational tension forces of the elastic thread depending on the parameters of the fibula and intramedullary blocking nail and on the location of the bone injury was obtained. The effect of foot rotation on the thread tension was investigated. The results of theoretical research should be implemented in medical practice.

**Conclusions:**

A mathematical model of the damaged fibula blocked by the intramedullary nail and fixed with the elastic thread was developed. Dependences for calculation of tension of the fixing thread were obtained. A slight increase in thread tension during foot rotation was found.

## 1. Introduction

Fractures of the lower extremities are a common type of injuries of human musculoskeletal system with the largest number of surgeries; the durations of treatment and functional recovery of the injured cause high rates of disability [1]. Modern medicine increasingly uses engineering solutions to improve and accelerate treatment. In traumatology, preference is given to a method of treatment, which provides rapid recovery of limb function [2].

Today, intramedullary attachments are a popular and widely used method of treating various fractures. Titanium nails are used for internal fixation of fractures of ulna [3], clavicle [4], tibia [5], and fibula [6] bones, as well as unstable fractures of ankle joints [7]. The work in [8] specified the prospect of intramedullary nails of small dimensions [9] instead of supraosseous plates to fix ankle fractures. The work in [10] compared biomechanically bionic, helical, and endobutton thread fixation during tibiofibular syndesmosis treatment. In present, there is no clear consensus on the optimum management of combined distal third tibia and fibula fractures [11–13].

The success of implant placement is evaluated by its long-term stability, which, in particular, is determined by the bone-implant interface biomechanical properties. Research [14] is devoted to alloy specification based on controlled training methods for biocompatible medical material designing. The paper [15] describes the design and engineering of implant manufacturing using additive technologies. The surfaces of biomaterials are subjected to various modifications to affect their physical and chemical properties as well as allow obtaining optimal surface topography [16], such as coatings on operational surfaces of implants [17–19]. These coatings improve surface properties and create effective compositions for combining different characteristics, such as strength, wear resistance, and blocking unwanted heat fluxes [20]. The authors also pay great attention to optimizing the structure of coatings [21] and study the behaviour of coatings with surface defects [22], features of crack propagation in coatings [23], and the possibility of effective healing of cracks [24].

A characteristic trend of recent years is the constant growth of the range and number of biomedical products that are manufactured by additive technologies. This branch of material production makes it possible to obtain new properties of products and save time and materials in their manufacture [25]. The additive manufacturing techniques allow creation of objects with complex shape as they are based on the process of joining materials, layer upon layer, differently from subtractive manufacturing methods [26]. Structural and mechanical properties play a crucial role in the design of biomedical devices with tailored performances which should satisfy the desired requirements. As an example, functional devices for tissue reconstruction should resemble the structure and properties of the natural tissue [27]. The control of the process-structure-property relationship of a material plays an important role in the design of biomedical metal devices featuring desired properties. The studies [28, 29] showed the possibility to directly act on the material-shape combination to modulate the mechanical behaviour of devices for different biomedical applications. Reverse engineering and additive manufacturing methods are required to achieve the design of customized devices with specific shape and size [30]. It is possible to avoid the effects of stress shielding and stress concentration. The 4D printed items will have the capacity to change the dimensions over the time, and it has well prospective for the biomedical field [31]. This article develops a mathematical model of fibula fracture blocked by biomedical products obtained by traditional methods. However, the approach developed by the authors may also represent an important starting point for future works aiming at a mathematical modelling in the case of advanced prosthesis.

From the point of view of modern biomechanics and medical engineering, the effects of contact interaction between the implant and biological tissues, as well as methods of reliable attachment of elements, are of interest [32, 33]. The work in [34] presents an analytical approach to simulate contact phenomena in a composition of two different materials; in particular, one of them has the features of biological structure, and the another one hasan artificial material with constant physical properties. Evaluation of the stress state of the bone tissue and contact stresses between the inner surface of the bone cavity and the implant is presented in [35].

Infections associated with implant placement have catastrophic consequences for patients. Voluminous and expensive works on wound treatment, implant removal, antibacterial therapy, and rehabilitation often accompany these cases. Nano-containing biopolymer film usage is a promising direction for accelerating wound healing [36].

However, some technical issues of stable-elastic fixation of ankle joint unstable fractures remain unresolved and require determination of clinical efficacy. The advantages of using intramedullary nails to provide fibula stable osteosynthesis and elastic fixation of the tibiofibular syndesmosis by threads and tape-coupler require mathematical biomechanical substantiation.

A number of issues remain debatable. The problems of necessity to provide a targeted blocking at different levels by intramedullary nails and three or four cortical insertion of a position screw, especially to fix fractures simultaneously with the destroyed distal syndesmosis, are still unsolved. Now, the tension force of the fixing thread for elastic contraction of syndesmosis is an off-protocol option determined subjectively by a surgeon. If the thread tension is too small, it will not perform its function. Excessive tension can create the danger of adverse deflections of the damaged fibula. This situation can lead to local stresses and deformations of bone tissues and secondary displacements of bone fragments, which will adversely affect the regeneration process.

There are almost no studies on the scientific substantiation aimed at specification of the fixing thread tension force for ankle joint unstable injuries of fibula trans- or suprasyndesmotic fractures (B, C Danis–Weber classification) and search for stress factors destabilizing stable-elastic fixation.

### 1.1. The Purpose of the Study

Determination of possible stress factors affects destabilization of the stable fibula osteosynthesis by the intramedullary nail with distal blocking and elastic fixation of distal syndesmosis by the thread with endobuttons by mathematical modelling of distal trans-and suprasyndesmotic unstable ankle injuries.

## 2. Materials and Methods

We used the bibliosemantic method and the content analysis, methods of structural-logical and system analysis. and methods of deformable solid mechanics for the research.

A mathematical conceptual model of unstable trans- and suprasyndesmotic fracture of the fibula (B, C Danis–Weber classification), stabilized by the intramedullary nail with distal blocking and damaged distal syndesmosis elastically fixed by the elastic thread with endobuttons, was developed. The intramedullary cylindrical nail had a hole perpendicular to the axis and located at an angle of 30° to the front plane of the nail and shin. Material of nail and endobuttons (CHARFIXsystem®) was titanium alloy. Elastic thread material (ARTREX® FiberWire®) No 5) was polyester.

We used the following mechanical properties of materials for numerical approbation of the research results. For bone tissue, modulus of elasticity, 17.9 GPa; Poisson's ratio, 0.3; strength limit, 125 MPa. For titanium intramedullary nail, modulus of elasticity, 112 GPa; Poisson's ratio, 0.32; yield strength, 250 MPa. For the fixing thread, modulus of elasticity, 1.45 GPa, and yield strength, 36 MPa. We theoretically specified the values of elastic thread tensile force, the fibula deflection, and the change in the thread tensile force during fibula displacement.

## 3. Results

### 3.1. Estimation of the Fibula Stiffness under the Influence of Localized Transverse Load

Figure 1 presents the tibia and fibula loading and fixing scheme. The main ideas of modelling are as follows. The stiffness of the fibula is much less than the stiffness of the tibia. The main contribution to the system flexibility during the tightening of the thread will make a change in the shape of the fibula due to the deformation of the bend. The fibula is placed in accordance with the rod of Figure 1(b). The tibia is considered absolutely rigid. The *lower* fibula-tibia connection (in the area of the foot) is modelled by a hinged movable support, and the upper connection (knee area) is modelled by a hinged fixed support. The concentrated force *P* schematizes the thread tension. It is necessary to specify a relation between the thread tension and linear and angular displacements of the fibula sections.

We introduce the Cartesian coordinate system *xow* (Figure 1(b)). The differential equation of the fibula deflections is as follows:

(1) $$\begin{array}{c} \frac{{\text{d}}^{2}w}{\text{d}x^{2}}=\frac{1}{E_{b}J}\left[\frac{P}{l}\text{bx}-P\left(x-a\right)\cdot H\left(x-a\right)\right], \end{array}$$

where *w* is the deflection of the fibula, *E*_*b*_ is the average Young's modulus of the bone tissues, *J* is the average axial moment of inertia of the fibula cross section, and *H*(*x*) is the Heaviside function. By twice integration of equation (1) and taking into account the boundary conditions [33, 37], we obtain expressions for determining the angles of rotation *ϑ*(*x*)=d*w*/d*x* and deflections *w*(*x*). Examining the expression of deflections to the extreme, we obtained a formula to specify the allowable force *P*=[*P*] at which the condition of stiffness of the fibula *w*_max_ ≤ [*w*] will be satisfied (maximum deflection *w*_max_ does not exceed the allowable value [*w*]).

The obtained expression (2) was made possible to specify the allowable value of the tension force of the fixing thread for the intact bone (Figure 1(b)):

(2) $$\begin{array}{c} \left[P\right]=9\sqrt{3}\frac{l}{b{\left(l^{2}-b^{2}\right)}^{3/2}}E_{b}J\left[w\right]. \end{array}$$

### 3.2. Assessment of the Damaged Fibula Stiffness Blocked by the Intramedullary Nail and Fixed with the Elastic Thread

Let us consider the fibula with the fracture blocked by the intramedullary nail, installed tightly in its channel. After that, the elastic thread with endobuttons fixes the broken fibula. This case of fibula reconstruction is modelled by a piecewise homogeneous rod with a surface with imperfection in the form of an ideal annular gap (Figure 1)(c). Part of the rod length of *t* has a tubular cross section; the other part of the rod length has a cross section in the form of bone tissue, titanium composition. We assume that, at the fracture site *x*=*s* (the area highlighted in Figure 1(c)) of the fibula which has completely lost its bearing capacity relative to the bend, only the intramedullary nail resists the transverse load.

Based on the aforementioned assumptions, we formulate the boundary problem of the piecewise homogeneous rod deformation, which simulates the fractured fibula (Figure 1(c)). We present the differential equation of displacements as follows:

(3) $$\begin{array}{c} \frac{{\text{d}}^{2}w_{i}}{\text{d}x^{2}}=\frac{1}{C_{i}}M_{i}\left(x\right),\;i=1,\ldots 4,\;x\in \left(0,l\right). \end{array}$$

where *C*_*i*_ is bending stiffness, *M*_*i*_(*x*) is the expression of the bending moment, *i* is thesite number (*i*=1, for 0 ≤ *x* ≤ *t*, *i*=2, for *t* ≤ *x* ≤ *a*, *i*=3, for *a* ≤ *x* ≤ *s*, and *i*=4, for *s* ≤ *x* ≤ *l*).

The integration of expression (3) leads to the eight constant integrations. Eight boundary conditions were used to find them:

(4) $$\begin{array}{c} w\left(0\right)=0,\\ w\left(l\right)=0,\\ w_{1}\left(t\right)-w_{2}\left(t\right)=0,\\ \frac{\text{d}w_{1}}{\text{d}x}\left(t\right)-\frac{\text{d}w_{2}}{\text{d}x}\left(t\right)=0,\\ w_{2}\left(a\right)-w_{3}\left(a\right)=0,\\ \frac{\text{d}w_{2}}{\text{d}x}\left(a\right)-\frac{\text{d}w_{3}}{\text{d}x}\left(a\right)=0,\\ w_{3}\left(s\right)-w_{4}\left(s\right)=0,\\ \frac{\text{d}w_{3}}{\text{d}x}\left(s\right)-\frac{\text{d}w_{4}}{\text{d}x}\left(s\right)=\left[\vartheta \right], \end{array}$$

where the jump of the angle of rotation [*ϑ*]=*ϑ*_3_ − *ϑ*_4_ at the fibula fracture area was found from the solution of the auxiliary problem. To study the fibula fracture behaviour, we considered a model in the form of two rigid blocks interconnected by an elastic layer (Figure 1(c)). The physical and mechanical properties of the elastic layer corresponded to the material properties of the intramedullary nail. This model was loaded with a bending moment *M*=*M*(*s*) equal to the bending moment at the fracture of the fibula. After examining the relationship between the applied moment and the angles of rotation of the blocks, we finally obtained

(5) $$\begin{array}{c} \left[\vartheta \right]=\vartheta_{3}-\vartheta_{4}=\frac{M\left(s\right)\Delta }{0.05d^{4}E_{t}}. \end{array}$$

Applying the scheme of the method of initial parameters [37, 38], the solution of problems (3)–(5) allows obtaining analytically a relation to determine the angles of rotation of the fibula cross sections *ϑ*(*x*)=d*w*/d*x* and an expression for deflections *w*(*x*). The obtained results are presented graphically. We have a system with the following parameters: *t*/*l*=1/2, *a*/*b*=7/3, *α*=4/11, *k*=2, and *s*/*l*=3/4.

Figure 2 shows the distribution of the angles of rotation of the cross sections along the length of the system. It is characteristic that the expressed angle point is present in the cross section; there is a change in the rigidity of the system (it is the point where the fibula tubular cross-section borders on the bone tissue-titanium composition cross section). A barely noticeable point of inflection is observed in the point of fibula loading with fixing thread, and there is an expressed jump of angles of rotation in the area of fibula fracture. The greater bending moment in the fracture area is associated with the jump of angles, besides the presence and magnitude of the jump depends on the gap between fibula fracture edges.

Figure 2(b) shows the distribution of deflections of the system. Comparing the graphical dependences 1 and 2, one can see that despite the inserted intramedullary nail, the fractured fibula was less rigid than the healthy bone. It should be noted that if the fracture is closer to the edge, the difference between the stiffness of the damaged and undamaged bones will decrease. On the deflection graphs, we observe the extrema, which correspond to the zero values of the angles of rotation of the cross sections. There is also a more expressed angular point at the fracture of the fibula. The greater the jump in the angles of rotation at the edges of the fracture is associated with, the more expressed the angular point is on the graph of transverse displacements.

Solving the problems (3)–(5), we obtained a formula for finding the allowable tensile strength of the thread *P*=[*P*], provided that the maximum deflection *w*(*x*^*∗*^)=*w*_max_ does not exceed the allowable value [*w*], and *x*=*x*^*∗*^ ≈ *l*/2 is the coordinate of the maximum deflection:

(6) $$\begin{array}{c} \left[P\right]=6\frac{C_{0}}{k}\frac{l}{b}\frac{\left[w\right]-1/2\vartheta_{0}l}{\left[1/8l^{3}+l-k/k\left(2t+1/2l\right){\left(t-1/2l\right)}^{2}\right]}. \end{array}$$

To apply expression (6), it is necessary to define a number of parameters and set the required values and constants:

(i) Angle of rotation for *x*=0:
  (7) $$\begin{array}{c} \vartheta_{0}=\frac{1}{C_{0}}\frac{Pb}{6l^{2}}\left[\left(1-k\right)t^{2}\left(3l-2t\right)+l\left(b^{2}-l^{2}\right)\right]+\left[\vartheta \right]\frac{l-s}{l}. \end{array}$$
(ii) Flexural stiffness of the fibula *C* and the fibula with the inserted intramedullary nail *C*_0_, respectively:
  (8) $$\begin{array}{c} C=0.05D^{4}\left(1-\alpha^{4}\right)E_{b},\\ C_{0}=0.05d^{4}E_{t}\left(1+\frac{E_{b}}{E_{t}}\frac{1-\alpha^{4}}{\alpha^{4}}\right),\\ \alpha =\frac{d}{D}. \end{array}$$
(iii) Young's moduli of the fibula *E*_*b*_ and the intramedullary nail *E*_*t*_ and their characteristic transverse dimensions *D* and *d*.
(iv) The stiffness ratio of the sections *k*=*C*_0_/*C* and the linear size *b*=*l* − *a*.

Let us consider two cases of admissible tension determination for the fixing thread for people of different heights; in both cases, we will consider variants of the damaged and undamaged fibula. We assumed the following numerical parameters:

- For the person of high height, *l*=0.37 m, *t*=0.19 m, *a*=0.31 m, *b*=0.06 m, *D*=0.011 m, *d*=0.004 m, and *s*=0.32 m
- For the person of low height, *l*=0.26 m, *t*=0.14 m, *a*=0.21 m, *b*=0.05 m, *D*=0.008 m, *d*=0.0035 m, and *s*=0.22 m

We draw the graphical dependences of the fibula maximum deflection [*w*] and refer to the tension force of the fixing thread (Figure 3). The vertical thick line marked the allowable deflection ([*w*]=0.003 m, for the person of high height, and [*w*]=0.002 m, for the person of low height).

The allowable deflection was specified from the condition of maintaining the geometrically correct shape of the fibula after growth (healing) of the fracture. If the actual deflection exceeds the permissible one, cracks or bone fracture edges may open, and the edges of the crack may be damaged upon contact, etc. The developed graphic dependences made possible definition of the admissible tension force of the elastic thread: if the person has high height (Figure 3(a)) [*P*]=32 *N* for the damaged fibula and [*P*]_0_=74*N* for the healthy one and if the person has low height (Figure 3(b)) [*P*]=17 *N* and [*P*]_0_=38 *N* accordingly. The shaded area (Figure 3) shows the zone of safe tension of the fixing thread during work with the damaged fibula.

### 3.3. Determination of the Additional Tension in the Fixing Thread Caused by the Fibula Movement Relative to the Tibia

If the foot rotates, there is a movement of the shinbones relative to each other. Let us determine how much the magnitude of the tension force in the fixing thread will change if the fractured fibula moves to the value of Δ_0_ relative to the tibia.

Using the model (Figure 4(a)), we jointly considered the static, kinematic, and biomedical aspects of the problem and obtained the formula for the additional force of tension of the thread *T*:

(9) $$\begin{array}{c} T=EF\frac{\sqrt{\Delta_{0}^{2}+a_{0}^{2}}-a_{0}}{a_{0}+\left(d_{0}+D\right)/\sqrt{{\left(\Delta_{0}/a_{0}\right)}^{2}+1}}, \end{array}$$

where *E* is Young's modulus of the thread material and *F* is the cross-sectional area of the thread. If the value (Δ_0_/*a*_0_)^2^ is a small value compared to one, then formula (9) can be written more compactly:

(10) $$\begin{array}{c} T=EF\frac{\sqrt{\Delta_{0}^{2}+a_{0}^{2}}-a_{0}}{a_{0}+d_{0}+D}. \end{array}$$

Figure 4(b) presents results graphically. The solid line shows the exact result (by formula (9)), and the dotted line shows the approximate result (by formula (10)). The additional tension of the thread *T* depends nonlinearly on displacement, and its growth rate increases with increasing the displacement. The stiffer thread for other equal conditions is associated with the greater additional tension. Comparison of solid and dotted curves indicates that we can use the approximate formula (10) if Δ/*a* < 0.4.

## 4. Discussion

Our proposed mathematical model allowed us to calculate an interaction of anatomical components, the shin. For practical application, the obtained results scientifically substantiate the tension magnitude of the thread, which reliably fixes the distal tibiofibular syndesmosis; the specified tension force will not create excessive displacement (deflection) of the bone fragments of the fibula.

Analytical calculations tested the hypothesis of the possible stress factor destabilizing the restored unstable injury of the ankle joint during the dosed load of the injured foot. Can excessive displacement (deflection) of the damaged fibula fixed by the intramedullary nail occur and, as a result, interfragmentary displacement due to local stresses? Can a change in the tension of the tape-coupler disrupt the matching of bone fragments due to multidirectional (axial, bending, extensor, and rotational) movements of the foot?

It was stated that the tension of the thread really increases slightly during the rotation of the foot. However, the amplitude of the anatomical mutual displacement of the tibia and fibula, stabilized by the tape-coupler, does not significantly affect the transverse and angular displacements of the damaged fibula, and it is not the stressor of secondary interfragmentary displacements and does not cause damage of the thread.

Specification of the rational thread tension during the stable-elastic fixation of through- and supra-syndesmosis fractures of the tibia will reduce the time of load starting of the injured limb, functional static and dynamic recovery of the patient in contrast to the method of rigid positioning of distal syndesmosis screw [10, 16]. Prolongation of treatment by this method is caused by the existing risk of destabilization, the risk of breaking the positional screw while walking, and the need for additional surgery to remove this screw.

In addition, the combined stable-elastic fixation allows avoiding large surgical incisions [9], which is especially important for the treatment of patients with ischemic manifestations of soft tissues due to trauma or comorbid pathology (diabetes, atherosclerosis obliterans, etc.). Besides, it allows predicting the effect of accelerating patient activation time by early dosed loading, which significantly reduces the time of functional recovery of the patient. In [39], it is noted that the application of elastic fixation will increase dynamically.

In further studies, it is planned to optimize the tensile strength of the thread, taking into account the contact of the fibula fracture edges.

## 5. Conclusion

1. The mathematical model of distal unstable injury of the ankle joint by stable fixation fibula fracture by the intramedullary nail as well as the obtained analytical dependences to determine the rational value of the tensile force of the elastic thread, which performs elastic fixation was developed.
2. We studied the effect of multivector displacement of the fibula which refers to the tibia on the value of the tensile strength of the elastic thread. It was found that the rotation of the foot, which causes additional load forces on the “fork” of the ankle joint, does not lead to a significant increase in thread tension.
3. The results of theoretical studies were put into the surgical practice for treatment of patients with trans- and supra-syndesmoses fractures of the fibula with damage to distal syndesmosis (44A3.2-A3.3, B2.1–B2.3, and C1.1–C3.3).

## Figures and Tables

**Figure 1:** The general view of tibia (a), the model of intact fibula (b), and the model of tibia with the fracture blocked by the intramedullary nail and fixed by the elastic thread (c).

**Figure 2:** Angles of rotation of cross sections (a) and deflections (b) of the fibula: 1 is the fractured bone blocked by the intramedullary nail and fixed with the elastic thread; 2 is the healthy bone loaded with fixing thread.

**Figure 3:** Determination of the fixing thread tension force for the stable-elastic fixation of unstable fractures of the ankle joint with damage to syndesmosis for the person of high height (a) and for the person of low height (b). 1 is the fractured fibula blocked by the intramedullary nail; 2 is the healthy fibula.

**Figure 4:** The model of fibula displacement during rotation of the foot (a) and the dependence of the additional tension in the fixing thread refer to displacement (b): 1–*d*/*a*=2/3and *D*/*a*=1 and 2–*d*/*a*=1 and*D*/*a*=2.

## Data Availability

All results obtained during the study are presented within the article.
